RETRACTED

# Efficacy and Safety of Minimally Invasive Transcatheter Closure of Congenital Heart Disease under the Guidance of Transesophageal Ultrasound: A Randomized Controlled Trial

**DOI:** 10.1155/2022/2969979

**Published:** 2022-07-14

**Authors:** Shuangyin Zhang, Xu Xu, Min Yu, Min Wang, Ping Jin

**Affiliations:** Department of Anesthesiology, Lanzhou University Second Hospital, Lanzhou 730030, China

## Abstract

**Objective:**

To investigate the efficacy of minimally invasive transcatheter closure of congenital heart disease (CHD) under the guidance of transesophageal ultrasound.

**Methods:**

A total of 100 patients with CHD treated in our hospital from February 2019 to April 2020 were enrolled in the group. The patients were randomly divided into control group and research group. The control group received minimally invasive transcatheter closure under the guidance of X-ray, and the research group received minimally invasive transcatheter closure under the guidance of transesophageal ultrasound. The operative results, the intraoperative- and postoperative-related indexes, and the incidence of early postoperative complications and follow-up results were compared.

**Results:**

First of all, we compared the results of the two groups: 48 cases of success, 2 cases of difficulty in the research group, 35 cases of success, 11 cases of difficulty, and 4 cases of failure in the control group. The success rate in the research group was higher than that in the control group (*P* < 0.05). Secondly, we compare the relevant indicators in the process of operation. The operation time, cardiopulmonary bypass time, upper and lower cavity obstruction time, and blood transfusion volume in the research group were lower than those in the control group (*P* < 0.05). In terms of postoperative-related indexes, the ventilator-assisted time, 24 h postoperative drainage, ICU time, and postoperative hospital stay in the research group were all lower than those in the control group (*P* < 0.05). The incidence of early postoperative complications in the research group was significantly lower than that in the control group such as secondary pleural hemostasis, pulmonary infection, pleural effusion, subcutaneous emphysema, poor incision healing, phrenic nerve loss, and right lower limb numbness (*P* < 0.05). All patients were followed up for 6 months, and the cardiac function of both groups returned to normal. There was no significant difference in the incidence of postoperative residual shunt and new tricuspid regurgitation. There was no significant difference in the data (*P* > 0.05). Considering abnormal ECG events, the incidence of abnormal ECG events (complete right bundle branch block, incomplete right bundle branch block, second- and third-degree block, left anterior branch block) in the research group was significantly lower than that in the control group (*P* < 0.05).

RETRACTED

**Conclusion:**

Minimally invasive transcatheter closure of CHD under the guidance of transesophageal ultrasound has the advantages of less trauma, less blood loss, short hospital stay, simple operation, less postoperative complications, and remarkable therapeutic effect. Minimally invasive transcatheter closure under the guidance of transesophageal ultrasound has the advantage of adapting to a wide range of syndromes and can be used for the closure of CHD in children. According to different types of CHD, registering the corresponding occlusive pathway can improve the success rate of operation. Through postoperative reexamination and regular follow-up, it is proved that minimally invasive transcatheter closure under the guidance of transesophageal ultrasound is safe, effective, and feasible.

## 1. Introduction

Congenital heart disease (CHD) refers to the abnormal development of the heart and blood vessels caused by various reasons during embryonic growth, including atrial septal defect (ASD), ventricular septal defect (VSD), and patent ductus arteriosus (PDA) [1]. There are many risk factors for CHD, which are not only genetic factors but also related to environmental, physical, chemical, and other factors [2]. It is generally believed that the occurrence of CHD is mostly the result of the joint action of environmental factors and genetic factors [3]. Critical and complex CHD newborns often indicate clinical manifestations such as cyanosis, shortness of breath, feeding difficulties, and repeated heart failure. If effective approaches of treatment are not taken, about 50% of the children will die during the neonatal period [4]. At present, CHD has become the main risk of neonatal death [5]. The incidence of CHD is high in China [6]. It has been reported that with the development of cardiac ultrasound and other techniques, the detection rate of congenital heart malformations such as micro ventricular septal defect and bicuspid aortic valve has been greatly increased, and the incidence of CHD in China can even reach up 75/1000 [7]. There are nearly 200 thousand new children with CHD in China every year [8]. In Europe and the United States, the fetal diagnosis rate of CHD can reach 20% ~47.3% [9]. It has become one of the major public health safety issues affecting the health and safety of the population and the quality of life in our country [10]. It has been reported that the preoperative condition of children with CHD diagnosed in fetal period is significantly better compared to neonatal period [11]. There are many kinds of CHD, which must be accurately and effectively diagnosed in time in order to provide protection for clinical treatment in the later stage. The general pathological types of CHD include VSD, ASD, atrio ventricular septal defect, pulmonary valve stenosis, and tetralogy of Fallot (TOF), especially VSD and ASD.

RETRACTED

The treatment of CHD includes surgical and medical interventional occlusion, as well as minimally invasive surgical occlusion which has sprung up in Chinese clinic in recent years [12]. At present, most heart clinical centers still treat CHD mainly by open chest repair under cardiopulmonary bypass (CPB) and interventional occlusion in internal medicine. The traditional surgical treatment of VSD and ASD is mainly direct vision repair of cardiac septal defect under CPB. With the increasing number of clinical cases of complex CHD, some traditional surgical treatments, especially in children with VSD, are subject to various limitations [13]. Moreover, conventional thoracotomy for open heart defect repair has the advantages of large trauma, long operation time, many postoperative complications, long hospitalization cycle, and high medical cost, which has been gradually eliminated in the treatment of simple CHD. With the advent of Amplatzer double disk occluder, interventional occlusion has become an important way to treat CHD [14]. It has been reported that transcatheter closure of CHD by medical intervention can significantly promote the cardiac function of patients with CHD, and the clinical effect is significant [15]. It is a common treatment for CHD at present. Although percutaneous catheter occlusion under medical X-ray is one of the effective clinical treatments for VSD and ASD, it is considered that X-ray has certain radiation damage to patients and surgeons. Especially for pediatric cardiac occlusion, it cannot be completed under nongeneral anesthesia digital subtraction angiography (DSA), which makes the clinical adaptation of interventional occlusion technique guided by DSA narrow, and then gradually replaced by minimally invasive surgical occlusion and eliminated [16]. In recent years, minimally invasive transcatheter closure of cardiac surgeons under the guidance of transthoracic or transfemoral artery or vein puncture under the guidance of esophageal echocardiography (TEE) has been increasingly carried out in China. This technique is favored by most cardiac surgeons and patients because of its unique green, safe, pollution-free, simple operation, less trauma, short operation time, and low medical cost. Minimally invasive surgical closure of VSD and ASD has become more mature after continuous technical improvement since it was employed in clinic. In this study, we focused on the efficacy and safety of transesophageal ultrasound-guided minimally invasive transcatheter closure of CHD.

RETRACTED

## 2. Patients and Methods

### 2.1. General Information

A total of 100 patients with CHD treated in our hospital from February 2019 to April 2020 were enrolled. The patients were randomly assigned into control group and research group. The control group received minimally invasive transcatheter closure under the guidance of X-ray, and the research group received minimally invasive transcatheter closure under the guidance of transesophageal ultrasound. In the control group, the age was 26-86 years old, with an average of 45.66 ± 2.37 years, including 27 males and 23 females, while in the research group, the age was 24-76 years old, with an average of 45.77 ± 2.64 years, including 26 males and 24 females. There exhibited no statistical significance in the general data between two groups (*P* > 0.05). This study was permitted by the Medical Ethics Association of our hospital, and all patients noticed informed consent.

Inclusion criteria are as follows: (1) there were no surgical taboos in blood routine and blood biochemical tests before operation; (2) ventricular and ASDs were diagnosed by TEE, and no other cardiovascular malformations were found [1–3]; (3) except for the subdry VSD, the other defects did not involve the adjacent heart valve; and (4) there was no more than moderate valvular regurgitation.

Exclusion criteria are as follows: (1) infectious disease within 2 weeks before operation, (2) mural thrombus in the cardiac cavity, (3) hemolytic disease or coagulation dysfunction, (4) patients with moderate or severe pulmonary hypertension (PAH) or Eisenmenger's syndrome, and (5) patients with decompensated heart failure and left ventricular ejection fraction (LVEF) < 30%.

### 2.2. Treatment Methods

The control group received minimally invasive closure under the guidance of X-ray, general anesthesia, and endotracheal intubation. The location, size, edge condition, and adjacent valve activity of the heart defect were evaluated, and the surgical minimally invasive closure was the same as the research group. The research group received transesophageal ultrasound-guided minimally invasive transcatheter closure, general anesthesia, and endotracheal intubation. The TEE probe was slowly placed in the esophagus, and the location, size, edge conditions, and adjacent valve activity of the defect were dynamically evaluated. Transthoracic closure: (1) median incision of 1.5 ~ 2 cm in the lower sternum, chainsaw split part of sternum, and xiphoid process; (2) incision and suspension of pericardium and intravenous injection of 1 mg/kg heparin; (3) transesophageal ultrasound guidance to locate the puncture point of heart surface; (4) double needle belt gasket and heart surface preset purse and puncture with cannula needle; (5) insertion of guide wire through defect; (6) sheath tube was placed along guide wire, and sheath core was removed; (7) choose the appropriate size occluder to release the left and right umbrella in turn; (8) after the occluder was released completely, the movement disturbance of the adjacent valve and the residual shunt around the defect were observed by ultrasound; (9) the steel wire was properly pushed and pulled to observe whether the occluder was firmly clamped; and (10) the steel wire and sheath were withdrawn. After successful transthoracic occlusion, tighten the purse and tie a knot with the surface of the heart, carefully stop the bleeding, close part of the pericardium, and routinely close the chest after indwelling the drainage tube. Percutaneous occlusion approaches: (1) femoral vein puncture and placement of 6F femoral sheath; (2) trans-vascular sheath insertion of 6F single curved catheter and rigid guide wire; (3) echocardiographic guidance of rotating catheter through the defect and placement of hard guide wire to the left superior pulmonary vein; (4) retention of guide wire and exchange of corresponding occluder transport sheath; (5) according to the diameter of the enrolled occluder, select the 718 F sheath; and (6) follow the guide wire into the left atrium and remove the sheath core. The follow-up steps are basically consistent with the transthoracic approach. After successful percutaneous occlusion, the puncture point was pressed to stop bleeding for more than 15 min. And after observing that there was no active bleeding at the puncture point, elastic bandage was applied and bandaged for 4 hours for 6 hours. All patients who received minimally invasive surgical closure were treated with 3 ~ 5 mg/kg aspirin for q.d.3 ~ 6 months, and the wound dressing was changed regularly during hospitalization. Echocardiography and electrocardiogram were reexamined at 1 month, 3 months, 6 months, and every year, respectively.

RETRACTED

### 2.3. Observation Index

#### 2.3.1. Surgical Results

According to the success of the operation, the surgical results are divided into three categories: (1) successful occlusion: the puncture point is accurate, the guide wire and guide sleeve pass smoothly, and the occluder is firmly clamped; (2) after the occluder is implanted, the guide wire and sheath are difficult to pass through the defect or do not match the diameter of the defect, so it is necessary to adjust the puncture point or replace the occluder to complete the occlusion. (3) Occlusion failure: occluder could not be implanted, adjacent valve activity disorder, atrioventricular block, and forced to give up occlusion.

#### 2.3.2. Related Indexes during and after Operation

Related indexes during operation are as follows: operation time, CPB time, blocking time of upper and lower cavity, and blood transfusion volume. Postoperative-related indicators are as follows: ventilator-assisted time, postoperative 24-hour drainage, ICU time, and postoperative hospital stay.

#### 2.3.3. Incidence of Early Postoperative Complications

The incidence of early postoperative complications such as secondary thoracic hemostasis, pulmonary infection, pleural effusion, subcutaneous emphysema, poor incision healing, phrenic nerve loss, and right lower limb numbness was calculated.

#### 2.3.4. Postoperative Follow-Up Results

The patients in the two groups were followed up for 6 months. The incidence of postoperative residual shunt and new tricuspid regurgitation was calculated. Meanwhile, the incidence of normal cardiac events (complete right bundle branch block, incomplete right bundle branch block, second- and third-degree conduction block, left anterior branch block) was calculated.

### 2.4. Statistical Analysis

The SPSS 22.0 statistical software is employed to analyze the data, and the data is based on statistics ± S.D.. It is indicated that *t*-test is employed for comparison between groups, counting data is expressed by example (percentage), and chi-square test is employed for comparison between groups. *P* < 0.05 indicates that the difference exhibits statistically significant.

## 3. Results

### 3.1. Comparison of Surgical Results

First of all, we compared the results of the two groups: 48 cases were successful, and 2 cases were difficult in the research group; 35 cases were successful, 11 cases were difficult, and 4 cases failed in the control group, and the success rate of the research group was higher compared to the control group (*P* < 0.05). All the data results are indicated in Figure 1.

### 3.2. Comparison of Related Indexes during Operation

Secondly, we compared the relevant indexes during operation. The operation time, CPB time, upper and lower cavity blocking time, and blood transfusion volume in the research group were lower compared to the control group (*P* < 0.05). All the data results are indicated in Table 1.

### 3.3. Comparison of Related Indexes after Operation

Thirdly, the postoperative-related indexes of the two groups were compared. The ventilator assist time, 24-hour postoperative drainage, ICU time, and postoperative hospital stay in the research group were lower compared to the control group (*P* < 0.05). All the data results are indicated in Table 2.

RETRACTED

### 3.4. Comparison of the Incidence of Early Postoperative Complications

Then, we compared the incidence of early postoperative complications. The incidence of early postoperative complications such as secondary thoracic hemostasis, pulmonary infection, pleural effusion, subcutaneous emphysema, poor incision healing, phrenic nerve loss, and right lower limb numbness in the research group was significantly lower compared to the control group (*P* < 0.05). All the data results are indicated in Figure 2.

### 3.5. Comparison of Postoperative Follow-Up Results

Next, we compared the postoperative follow-up results of the two groups, and all patients were followed up for 6 months successfully, and the cardiac function of the two groups returned to normal after operation. There exhibited no significant difference in the incidence of postoperative residual shunt and new tricuspid regurgitation (*P* > 0.05). All the data results are indicated in Table 3.

### 3.6. Comparison of Abnormal ECG Events

Finally, we compared the abnormal ECG events. The incidence of abnormal ECG events (complete right bundle branch block, incomplete right bundle branch block, degree II and III conduction block, left anterior branch block) in the research group was significantly lower compared to the control group (*P* < 0.05). All the data results are indicated in Table 4.

## 4. Discussion

CHD seriously affects the physical and mental health of infants [15]. VSD is the most common CHD, accounting for about 25% of the total. Perimembranous ventricular septal defect is the most common type of ventricular septal defect, accounting for about 80% [16]. At the later stage of the disease, there are more complicating diseases, especially when the defect becomes larger and larger, which leads to a significant increase in left ventricular volume load, with varying degrees of fatigue, shortness of breath, pulmonary hypertension, cardiac dysrhythmia, and other symptoms and finally evolves into Eisenmenger syndrome, that is, irreversible right-to-left shunt [17]. Therefore, once the disease is diagnosed, it needs to be treated immediately. The traditional treatment of VSD is open thoracotomy under CPB. However, this technique requires median sternal incision, great trauma, more bleeding during operation, slow recovery after operation, CPB and transfusion of blood products, and potential complications of CPB after operation, such as cognitive dysfunction, coagulation disorder, and renal dysfunction [18]. The healing deformity after sternotomy and the incision scar located in the middle of the chest can cause psychological disorders and affect the long-term quality of life of the patients. Percutaneous interventional occlusion of VSD in internal medicine was first completed by van Egmond Dam et al. in the 1970s [18]. Due to its minimally invasive and beautiful incision, it is widely accepted [17, 18]. However, percutaneous intervention in the department of internal medicine needs to be completed under the guidance of radiation, which can cause inevitable damage to doctors and patients, and it has been proved that long-term radiation irradiation has carcinogenic effect. Transthoracic minimally invasive transcatheter closure is a new hybrid technique which integrates internal and surgical techniques. In 2007, Marwali Eva et al. first carried out minimally invasive transcatheter closure of membranous VSD under the guidance of ultrasound, transsternal segment, and non-CPB [19]. This technique avoids the shortcomings of CPB and significant trauma repaired by surgery and radiation injury caused by percutaneous interventional therapy in internal medicine. However, this technique shortens the surgical incision and sternotomy on the basis of surgical sternotomy, but the trauma of sternotomy, poor sternal healing, and incision scar in the presternal area still exist, which will still cause psychological disorders and affect the long-term quality of life of patients [20].

RETRACTED

At present, the treatment of CHD mainly includes traditional thoracotomy, percutaneous catheter closure, minimally invasive surgery with various small incisions, video-assisted thoracoscopic surgery, and robot-assisted surgery [21]. Although surgical thoracotomy and direct vision defect repair under CPB are not affected by the patient's age, body weight, and defect diameter and location, especially for young age, low body weight, and complicated with pulmonary hypertension, even patients with failed interventional occlusion have absolute advantages [22]. However, there are some shortcomings in the above treatments: (1) median thoracotomy and CPB in traditional surgery will cause great trauma to the patient's body, accompanied by increased intraoperative blood loss, slow postoperative recovery, unpleasant incision healing, and especially great influence on postoperative respiratory function in high-risk patients; (2) video-assisted thoracoscopic and robot-assisted surgery systems require special equipment and long-time learning to master complex operations; (3) percutaneous catheter interventional occlusion should be performed under the guidance of DSA, which causes damage to patients and surgeons to a certain extent, and once the closure fails, it is difficult for cardiologists to achieve thoracotomy repair under CPB. Many shortcomings narrow the clinical adaptation syndromes of the above various treatment methods of CHD [22–25]. Minimally invasive surgical closure integrates the related advantages of open-heart defect repair and percutaneous catheter closure under CPB, avoids the shortcomings of various surgical procedures, and shows the advantages of rapidness, convenience, strong applicability, flexible operation, and complementary internal and surgical procedures. Meanwhile, it can minimize the risk of operation, avoid the injury caused by X-ray and catheter intervention, improve the curative effect of operation, and effectively reduce the incidence of various complications [26, 27].

RETRACTED

The American Echocardiography Association recommends transesophageal echocardiography for preoperative diagnosis and guidance of transcatheter closure of ASD [26]. Compared with TEE, the imaging effect of TEE is better; the ultrasonic probe stays in the patient's esophagus, which is adjacent to the heart, which avoids the interference of pneumonic lungs to the imaging effect, especially in the observation of the structure of the posterior part of the heart near the esophagus [27]. Minimally invasive closure of cardiac surgery generally chooses transesophageal echocardiography to guide the guide wire and transport sheath through the defect and participating in the transport and release process of the occluder and the effect of real-time dynamic feedback [28]. The complications such as the opening and closing of the surrounding valve and the residual shunt after the closure of the defect were observed immediately after the operation, which provided a direct and objective basis for the evaluation of the effect of the operation [28]. In minimally invasive transcatheter closure of CHDs such as VSD, ASD, and PDA, TEE is the eye of surgeons, which can effectively guide surgeons to successfully block all kinds of CHDs, which is the key in the whole operation [29]. Transesophageal ultrasound-guided minimally invasive transcatheter closure has two surgical pathways: transthoracic and percutaneous occlusion. Transthoracic approach can clearly show the tissue structure of the heart without blocking the visual field of the operation, and the complete puncture process can be monitored dynamically. Transesophageal ultrasound can evaluate the disturbance of adjacent valve activity and III degree atrioventricular block after occluder implantation and a series of advantages such as immediate conversion to thoracotomy to save patients when the occluder fails or the occluder falls off [29, 30]. It is generally considered as the preferred occlusion path for VSD or ASD with larger defect diameter; percutaneous closure is often used in pediatric ASD because of no X-ray, no pollution, no chest incision, less blood loss, more minimally invasive, and supported by surgery [30]. However, there are still some weaknesses in percutaneous occlusion, including long operation path, strict mastery of intravascular sheath and guide wire operation skills, long learning curve of physicians, and blind area of visual field in a certain area in the process of ultrasound-guided transcatheter closure [31].

RETRACTED

Considering the findings of other scholars [32–34], (1) the success rates of percutaneous closure of small aperture (defect diameter ≤ 5 mm) ASD and transthoracic closure of defect diameter ≤ 10 mm ASD were both 100%; (2) the small aperture ASD is mainly central type, and the guide wire and sheath may be occluded by secondary septum during transthoracic closure, and the success rate is higher because the forward direction of the guide wire and sheath is at an angle to the defect opening during percutaneous closure; (3) for the ASD with defect diameter 6 mm~20 mm, the two occlusion paths are available, and there is no statistical difference in success rate, but percutaneous closure is more minimally invasive. It is particularly important to adjust the release angle of the occluder during percutaneous transcatheter closure of ASD. Meanwhile, be aware of the rupture caused by violent traction of the guide wire into the left atrial appendage; (4) the transthoracic closure effect of transthoracic closure under the guidance of transesophageal ultrasound is better for the ASD of defect diameter 21 mm~35 mm. Because the transthoracic closure is more direct, there is no blind area in the ultrasonic imaging operation, and the surgical field of vision is more intuitive. Relatively speaking, percutaneous closure is rarely adopted because of the difficulty of vascular dilatation; the guide wire and sheath cannot be vertical defect plane, resulting in the increase of parachute replacement rate, closure difficulty, and the probability of failure; (5) for the ASD with defect diameter > 35 mm and good defect edge condition, the transthoracic approach with short operation path and good occluder release angle is generally chosen. Even so, the difficulty of occlusion and the possibility of failure of occlusion are significantly higher than those of ASD patients with defect diameter ≤ 35 mm, and it is very likely that the occluder is attached or clamped unfirmly because the defect diameter is too large, resulting in the loss of the occluder after operation [35]. Our research results are consistent with the above conclusions, which shows that this study has good value.

RETRACTED

Our study still has some limitations. First of all, the trial only included 100 cases, and the number of the patients could influence the results of our investigation. We will continue to expand our case number and do even long-term follow-up of previous study participants. In addition, our study was constrained by a number of interventions and applicable criteria. The subjects selected for the study are not representative enough, to the extent that they may affect the experimental results to varying degrees.

In summary, transesophageal ultrasound-guided minimally invasive transcatheter closure of CHD has the advantages of less trauma, less blood loss, short hospital staying, simple operation, less postoperative complications, and remarkable therapeutic effect. Transesophageal ultrasound-guided minimally invasive transcatheter closure has the advantage of adapting to wide syndrome and can be employed in the closure of CHD in children. According to different types of CHD, the corresponding occlusion path should be enrolled, which can promote the success rate of operation. Through postoperative reexamination and regular follow-up, it is proven that transesophageal ultrasound-guided minimally invasive transcatheter closure is safe, effective, and feasible.

## Figures and Tables

**Figure 1:** Comparison of surgical results between two groups.

**Figure 2:** Comparison of the incidence of early postoperative complications between two groups.

**Table 1:** Comparison of intraoperative-related indexes between the two groups ($\bar{x}\pm s$).

Grouping	*N*	Operation time (min)	CPB time (min)	Upper and lower cavity blocking time (min)	Blood transfusion volume (ml)
Control group	50	154.85 ± 23.52	68.93 ± 3.76	38.59 ± 9.42	389.81 ± 24.77
Research group	50	142.55 ± 14.32	51.58 ± 3.55	28.39 ± 10.21	294.82 ± 25.55
*t*		3.158	23.724	5.191	18.874
*P*		<0.05	<0.05	<0.05	<0.05

**Table 2:** Comparison of related indexes after operation between the two groups ($\bar{x}\pm s$).

Grouping	*N*	Ventilator assist time (min)	Drainage 24 hours after operation (ml)	ICU time (h)	Postoperative hospital stay (d)
Control group	50	14.54 ± 2.42	386.93 ± 26.23	44.93 ± 8.31	14.29 ± 2.12
Research group	50	8.82 ± 1.44	273.91 ± 25.33	27.39 ± 4.21	6.58 ± 1.22
*t*		14.362	21.916	13.313	22.288
*P*		<0.05	<0.05	<0.05	<0.05

**Table 3:** Comparison of postoperative follow-up results between the two groups (*n*/%).

Grouping	*N*	Residual shunt		New tricuspid regurgitation	
		3 months	6 months	3 months	6 months
Control group	50	3 (6.00)	4 (8.00)	5 (10.00)	2 (4.00)
Research group	50	1 (2.00)	1 (2.00)	1 (2.00)	1 (2.00)
*χ* ^2^		1.041	1.894	2.836	0.343
*P*		>0.05	>0.05	>0.05	>0.05

RETRACTED

**Table 4:** Comparison of abnormal ECG events between the two groups (*n*/%).

Grouping	*N*	Complete right bundle branch block	Incomplete right bundle branch block	Second- and third-degree conduction block	Left anterior branch block	Total incidence rate
Control group	50	4 (8.00)	5 (10.00)	5 (10.00)	4 (8.00)	18 (36.00)
Research group	50	2 (4.00)	2 (4.00)	2 (4.00)	1 (2.00)	7 (14.00)
*χ* ^2^						6.453
*P*						<0.05

## Data Availability

The datasets used and analyzed during the current study are available from the corresponding author upon reasonable request.
